The article "Antibiotic Resistance Knowledge, Attitudes, and Practices among Pharmacists: A Cross-Sectional Study in West Bank, Palestine" was published in 2023. Journal: J Environ Public Health.

# Antibiotic Resistance Knowledge, Attitudes, and Practices among Pharmacists: A Cross-Sectional Study in West Bank, Palestine

**DOI:** 10.1155/2023/2294048

**Published:** 2023-01-30

**Authors:** Diala Abu Al-Halawa, Rania Abu Seir, Radwan Qasrawi

**Affiliations:** ^1^Faculty of Medicine, Al-Quds University, Jerusalem, State of Palestine; ^2^Faculty of Science and Technology, Al-Quds University, Jerusalem, State of Palestine; ^3^Department of Computer Engineering, Istinye University, Istanbul 34010, Turkey

## Abstract

Antibiotic resistance is an increasing problem worldwide. Dispensing antibiotics without prescription is a major contributing factor to antibiotic resistance. Pharmacists as healthcare providers are, in many studies, considered responsible for this practice. This study aims to explore Palestinian pharmacists' knowledge, attitudes, and practices concerning antibiotic resistance. A descriptive cross-sectional survey was conducted in 2021–2022. A random sample of 152 pharmacists was selected from the West Bank. Data were collected using a self-administered questionnaire that includes five sections: demographic characteristics, knowledge, attitudes, practices, and potential interventions. Results indicated that 60% of pharmacists dispense antibiotics without a prescription. A significant association between pharmacies' locality and antibiotic knowledge, attitudes, and practices was found. Pharmacists' knowledge-related responses indicated that 92.1% of the pharmacists agreed that inappropriate use of antibiotics can lead to ineffective treatment and 86.2% disagreed that patients can stop taking antibiotics upon symptoms' improvement. Only 17.1% disagreed that antibiotics should always be used to treat upper respiratory tract infections. Over two-thirds considered that they are aware of the regulations about antibiotic dispensing and acknowledged that antibiotics are classified as prescription drugs. Furthermore, 71.7% and 53.3% agreed that they have good knowledge of the pharmacological aspects of antibiotics and antibiotic resistance. Concerning attitudes, 75.6% agreed that antibiotic resistance is an important and serious public health issue facing the world, and 52% thought that antibiotic dispensing without a prescription is a common practice in the West Bank. Our findings indicate that pharmacists' locality and practices related to antibiotic dispensing without prescription are associated with the increase in antibiotics misuse and bacterial resistance. There is a need to design education and training programs and implement legislation in Palestine to decrease antibiotic resistance.

## 1. Introduction

Antibiotic resistance is becoming a global public health issue due to the increased morbidity, mortality, and healthcare costs attributed to resistant bacteria [1–4]. Antibiotic-resistant bacteria have become a serious threat. At the global level, more than 700,000 deaths are caused by antibiotic-resistant bacteria each year, and it is estimated that the number of deaths could grow to 10 million deaths per year in 2050 [5].

Irrational antibiotic use including overuse, suboptimal use in terms of dose and duration, and use with the wrong indication exacerbates the phenomenon [4, 6, 7]. Access to nonprescription antibiotics is a crucial factor related to this irrational use, as over 50% of antibiotics worldwide are purchased without prescription [8, 9]. Due to the rising issue of antibiotic resistance, numerous researchers have studied the contribution of the healthcare providers to this problem. Pharmacists, as key dispensers of antibiotics, could be major contributors to antibiotic resistance in Palestine and the world [10–13]. In Saudi Arabia, 98% of pharmacies reported dispensing antibiotics without prescription [6, 14]. Another study showed that the pharmacy was the main source of antibiotic self-medication (>90%) [15]. Although these results emphasize the importance of addressing pharmacists' reasons behind dispensing antibiotics without prescription, a multitude of factors could affect pharmacists' practices including their knowledge and attitudes towards antibiotic resistance. Lack of current knowledge about indications and uses, fear of loss of customers to competing pharmacies, and low level of adherence to existing legislation are some contributing factors, to name a few [16–21].

Despite the legislations the Palestinian Ministry of Health issued regarding dispensing antibiotics without prescription, antibiotic overuse increased due to the lack of sufficient application of the regulations and the availability of antibiotics in the private market without prescription [22]. Consequently, it is important to investigate the role of pharmacists in antibiotic resistance in the Palestinian community, as their knowledge, attitudes, and practices have a significant association with antibiotic misuse and overuse globally. Therefore, this study sought to assess the knowledge, attitudes, and practices of Palestinian pharmacists towards antibiotic resistance, as a basic ground for legislations and public health initiatives to tackle this ever-growing problem.

## 2. Materials and Methods

### 2.1. Study Design and Sampling

A descriptive cross-sectional survey was conducted among Palestinian pharmacists between October 2021 and February 2022 to assess their knowledge, attitudes, and practices towards antibiotic resistance. Participants with a minimum of two-year work experience in pharmacy were selected. All participants only had either at least a bachelor's degree in pharmacy or Pharm D. A random sampling approach was used through a three-step sampling method to ensure generalizability and minimize selection bias. First, the total number of registered community pharmacies in the West Bank (1084 pharmacies) was determined [23]. Next, a representative sample of 167 pharmacies was selected from the sample frame using the following random sampling parameters (15% of the population size; confidence level = 95%; margin of error = 5%). Random pharmacies were approached from the West Bank, and out of each pharmacy, one pharmacist was included in the survey.

### 2.2. Study Tool

A validated self-administered questionnaire was developed based on a thorough literature search through web-based databases and related studies [24–26]. The initial version of the questionnaire was developed in the English language and the final version was translated into Arabic language. The translation was validated using the standard forward-backward method [27]. The validation of the study instrument was performed by six experts, including two researchers, a pharmacologist, a clinician, a pharmacist, and an expert from the Palestinian Ministry of Health. In addition, the study was pilot tested on 20 pharmacists. The study instrument was modified based on the experts' comments and pilot test results. A final version was released and used for the data collection.

### 2.3. Measures

The final data collection instrument included questions to assess the sociodemographic characteristics of respondents, 19 questions to assess knowledge, 6 questions to assess attitudes, 10 questions to assess practices, and 3 questions regarding the potential interventions of the respondents towards antibiotic resistance.

The sociodemographic characteristics include gender, geographical location, education, type of employment, working hours, the total number of employed pharmacists, the number of working pharmacists at once in the pharmacy, and years of experience.

The knowledge assessment scale of 19 items using a Likert scale of 5 to 1 (5: strongly disagree, 4: disagree, 3: neutral, 2: agree, and 1: strongly agree) was used to assess the pharmacists' knowledge about antibiotics and antibiotic use, antibiotic resistance, legal aspects of antibiotic dispensing, and self-perception of their knowledge level.

Attitudes were assessed by an 8 items' scale using a Likert scale of 5 to 1 (5: strongly disagree, 4: disagree, 3: neutral, 2: agree, and 1: strongly agree). In addition, the section included a multiselection subsection on contributing factors to antibiotic resistance.

The practices were assessed by a 6 items' scale using a Likert scale of 5 to 1 (5: never; 4: rarely; 3: sometimes; 2, often; and 1, always). Practices section also included three questions on the total number of dispensed antibiotics per day, the number of dispensed antibiotics per day with prescription, and the number of demanded antibiotics without prescription per day. Furthermore, the section included a multiselection subsection for sources of information used as guidelines/references for antibiotic dispensing.

The negative statements were reverse scored during the analysis, and the responses to the knowledge, attitudes, and practices Likert scale questions were summed, so that higher scores reflect a positive direction towards antibiotic resistance, respectively.

A Cronbach's alpha test was conducted to assess the internal reliability of the questionnaire: the alpha scores were 0.75 and 0.745 for knowledge and attitudes indicated moderate reliability for these sections, and an alpha score of 0.859 for practices indicated high reliability for the practices' questionnaire, respectively.

Furthermore, three questions related to potential interventions, and the role of involvement in educational seminars about antibiotic resistance was included in the data collection instrument.

### 2.4. Data Collection

The data were collected under the supervision of the Ministry of Health and Al-Quds University. Six trained field researchers who had received training in conducting field research visited the selected community pharmacies. They were provided with a data collection guideline. Before completing the study questionnaire, the study objectives were explained to participants and consent to participate in the study was obtained. Overall, 167 participants agreed to participate in the study, and 152 completed the questionnaire.

### 2.5. Statistical Analysis

Data were coded, entered, cleaned, and analyzed using SPSS version 21.0 software (SPSS Inc., Chicago, IL, USA). Descriptive statistics (frequencies and percentages) were used to summarize the data. The chi-square, univariate, and linear regression analysis were used, where indicated, to assess the relation between demographic characteristics and knowledge, attitudes, and practices towards antibiotic resistance. A *p* value of less than 0.05 was considered statistically significant.

## 3. Results

### 3.1. Demographic Characteristics of Respondents

Out of 167 questionnaires distributed, 152 participants (91.01%) completed the survey. The study participants consisted of 52% females and 48% males, and 50.7% aged <30 years. Around 51.3% of the participants resided in rural areas. A 40.8% of them had at least 10 years of experience, and 75.3%, 14.4%, and 10.3% had a bachelor's, postgraduate, and Pharm D degrees, respectively. Furthermore, around 64.5% were employees in their pharmacies, while the rest were managers. In addition, 71.1% of the pharmacists reported working part-time, and only 28.3% had a full-time workload. Around two-thirds of the pharmacies had up to 3 employed pharmacists and one pharmacist working at once (59.9% and 62.5%, respectively). The demographic and professional characteristics of the participants are shown in Table 1.

### 3.2. Knowledge of Antibiotic Resistance

The knowledge of Palestinian pharmacists regarding antibiotic use and antibiotic resistance were assessed using the knowledge scale. Most of the pharmacists agreed that inappropriate use of antibiotics could lead to ineffective treatment (92.1%). When asked about general antibiotic use, around 72% of the pharmacists disagreed that antibiotics could be used to alleviate pain. Furthermore, 86.2% disagreed that patients could stop taking antibiotics when their symptoms improved, and 66.5% acknowledged that keeping leftover antibiotics for use in another time was not a good practice. Interestingly, only 17.1% disagreed that antibiotics should always be used to treat an upper respiratory tract infection. Concerning antibiotics' side effects, two-thirds of the participants knew that antibiotics could kill normal flora in the body, thereby causing secondary infections, and around 83% agreed that antibiotics could cause allergic reactions. Regarding certain common medications, surprisingly, around 9% disagreed that amoxicillin is an antibiotic. In addition, around 6% agreed that Panadol and aspirin are antibiotics, and 6.6% were uncertain.

Concerning knowledge of antibiotic resistance, around 42% of the participants thought that prescribing broad-spectrum antibiotics is always better, despite the possibility of available narrow-spectrum antibiotics. When asked about the mechanism of resistance of certain types of bacteria, around 70% knew that the mechanism of resistance to beta-lactams in *Klebsiella pneumoniae* is mainly enzymatic, while around 42% were uncertain of the mechanism of resistance in vancomycin-resistant *Enterococcus faecalis*. However, over two-thirds agreed that the wrong choice of antibiotics may lead a pathogen to lose its sensitivity towards a specific antibiotic, and that skipped antibiotic doses contributed to the development of antibiotic resistance. Additionally, around 40% thought that resistant bacterial strains could be spread in healthcare facilities.

When asked about their knowledge of antibiotic dispensing without prescription, over two-thirds considered that they were familiar with the rules concerning the dispensing of antibiotics (with or without a prescription) in the West Bank and acknowledged that antibiotics are classified as prescription drugs. Furthermore, when asked about their perception of their own knowledge regarding antibiotic uses and resistance, 71.7% and 53.3% agreed that they have good knowledge of the pharmacological aspects of antibiotics and of antibiotic resistance, respectively.  Table 2 shows results of questions about knowledge of antibiotic uses and antibiotic resistance.

### 3.3. Attitudes towards Antibiotic Resistance

The attitudes section is comprised of questions within four conceptual categories: antibiotic dispensing, pharmacist/patient interaction related to antibiotic resistance, required education concerning antibiotic dispensing and resistance, and major contributing factors to antibiotic resistance. Result in Table 3 indicates that most of the pharmacists agreed that antibiotic resistance is an important and serious public health issue facing the world (75.6%). As for antibiotic dispensing, 52% thought that antibiotic dispensing without a prescription was a common practice in the West Bank, while 36.2% were uncertain. Concerning interaction with patients, 63.8% of the pharmacists tried to educate patients when they asked for antibiotics without a prescription.

The pharmacists were asked about the importance of education programs related to antibiotic use and resistance. Around 70.2% concurred that they are in need of attending educational programs to enhance their understanding of antimicrobial stewardship. In addition, around 52.6% indicated that the development of local guidelines would be more useful than the international guidelines.

Figure 1 shows the pharmacists' responses towards the factors most likely contributing to the increase of antibiotic resistance. Results showed that related to patients, the most important contributing factors are the use of antibiotics without a prescription (66.4%) and patient noncompliance with the proper use of antibiotics (65.1%). Furthermore, 46.7% and 40% thought that patients' insistence on purchasing antibiotics and improper patient education contributed to the issue. Concerning health professionals, the participants reported that pharmacists' improper antibiotic dispensing (52%), and physicians' improper prescription practices (41.4%) are important factors contributing to antibiotic resistance. In addition to the above factors, 36.8% thought that illegal marketing practices added to the problem.

### 3.4. Practices towards Antibiotic Resistance

The results in Table 4 shows the number and percentage of antibiotic packets dispensed and demanded per pharmacy per day. 57.8% of the pharmacists reported up to 20 antibiotic sales per day, whereas 38.8% dispense over 20 antibiotics per day. Most of their dispensed antibiotics were with prescription only (77.6%). Furthermore, most of the pharmacists' reported that they encounter under 20 antibiotic demands without prescription (90.8%).

Table 5 presents the results of practices-related questions. Concerning antibiotic dispensing: 26.3% always, 8.6% often, and 25% sometimes of the pharmacists dispensed antibiotics without a prescription; one-third sold them for adults with recognized minor bacterial infections (2.6% always and 29.6% often); and 21.7% always and 15.1% often dispensed antibiotics without prescription for known customers. Moreover, the participants reported encouraging patients to obtain a physician's consultation and get a prescription (37.5% always and 22.4% often), while around two-thirds reported that they asked about drug allergies and health problems before dispensing antibiotics without a prescription (55.9% always and 11.8% often), and 29.6% always, and 17.8% often of them warned about their potentials side effects and educated patients on proper antibiotic usage (35.5% always and 22.4% often). Additionally, 16.4% always and 20.4% often seek additional clinical information before dispensing antibiotics without a prescription.

Figure 2 shows the percentage of pharmacists' responses to some of the possible reasons for dispensing antibiotics. Most of them reported selling due to patients' refusal to consult the physician unless they were seriously ill (67.1%) or patients' inability to afford the physician's consultation fee (58.6%), and 32.2% believe that pharmacists' good knowledge was a possible reason. In addition, 40.1% reported fear of losing their customers, whereas around one-third reported lack of awareness of the regulations that prohibit dispensing without a prescription. Regarding financial profits, around one-third reported that the pharmacy's owner's insistence to maximize the profits and fear of getting in trouble for refusing to sell over the counter antibiotics compelled them to sell without prescription.

Around 68% of participants referred to WHO guidelines, and 50.7% of participants reported the use of international guidelines as sources for antibiotic dispensing practices. Only 14.5% of participants used the national guidelines of the Palestinian General Directorate of Pharmacy's guidelines as a reference. Over half of the participants reported the use of the Internet (55.9%) and medical journals (25%), while others obtained information from senior, experienced colleagues and physicians (42.8% and 28.3%), respectively.

### 3.5. Potential Interventions

When the participants were asked about their attendance at workshops on antimicrobials, only 17.8% reported having some training on the use of antibiotics. Moreover, 89.5% expressed their desire to acquire further education and training on antimicrobial use, resistance, and stewardship. Most of the pharmacists reported they would like to attend workshops and training programs (67.1%). Whereas fewer participants expressed their desire to participate as consultants (15.1%), developers of courses (12.5%), mentors to other pharmacists (9.9%) and leader of workshops and stewardship programs (4.6%).

### 3.6. Knowledge, Attitudes, and Practices Scores

The overall pharmacists' knowledge, attitudes, and practices were estimated by summing the scales items scores. The overall mean knowledge score was 69.2 (SD = 8.41; range = 43; maximum possible score = 87), and the mean attitudes score was 27.3 (SD = 4.61; range = 27; maximum possible score = 35), whereas the mean practices score was 39.3 (SD = 8.18; range = 130; maximum possible score = 55). Linear regression analysis was performed to assess for associations between the knowledge, attitudes, and practices' scores and demographic variables.  Table 6 presents the results of the association between of the sociodemographic variables and the above-mentioned scores. Concerning knowledge, the results demonstrate significant associations with gender, locality, and number of employed pharmacists (*p* = 0.014; *p* = 0.001; *p* = 0.001), where females (OR = 1.23; 95% CI = 0.94–8.15), those living in urban areas (OR = 1.55, 95% CI = 6.39–12.66) are more likely to have a higher knowledge score, and workers in pharmacies with a higher number of employees are more likely to have a lower knowledge score (OR = 0.76; 95%CI = −9.7 to −2.67). The results showed no statistically significant effect of the number of working pharmacists at once (*p* = 0.736), education (*p* = 0.807), employment type (*p* = 0.540), age (*p* = 0.792), or years of experience (*p* = 0.988) on the knowledge score, however, pharmacists who are employees rather than managers and older pharmacists are 1.05 (95% CI = 05.03) and 1.03 (95% CI = 0–6) times likely to have slightly higher knowledge score, respectively.

As for attitudes score, the results showed no significant association with education level (*p* = 0.005), locality (*p* = 0.005; *p* = 0.001), gender (*p* = 0.296), total number of employed pharmacists (*p* = 0.321), number of employed pharmacists working at once (*p* = 0.312), employment type (*p* = 0.926), age and years of experience (*p* = 0.385; *p* = 0.773), respectively. However, pharmacists with a higher educational level and older pharmacists are 1.15 (95% CI = 0–1.87) and 1.17 (95% CI = 0–1.77) times more likely to have a higher attitude score, respectively. Female pharmacists, pharmacists who work in pharmacies with a larger staff, and those living in urban areas are 1.10 (95% CI = 0–2.3), 1.03 (95% CI = 0–1.72), and 1.08 (95% CI = 0–1.98) more likely to have better attitudes, respectively.

Finally, the results of the practices score association with the demographic variables demonstrated that there was a significant association with the number of employed pharmacists and locality (*p* = 0.001; *p* = 0.001). The pharmacists working in pharmacies with a higher number of employees reported lower practices score (OR = 0.74; 95% CI = −7.72 to −2.42), however those living in urban areas are more likely to have higher practices score (OR = 1.50, 95% CI = 4.49 –9.02). However, there were no significant differences in the practices score by gender (*p* = 0.191), number of employed pharmacists working at once (*p* = 0.498), employment type (*p* = 0.919), age (*p* = 0.121), and years of experience (*p* = 0.337). The odds of having a higher practices score are observed in females (OR = 1.12; 95% CI = 0–4.52), more educated pharmacists (OR = 1.1; 95% CI = 0–3.05), and more experienced pharmacists (OR = 1.14, 95% CI = 0–6.52).

## 4. Discussion

This current study reflects on the initial understanding of pharmacists' perspectives and role in antibiotic resistance in Palestine, as one of the low- and middle-income (LMIC) countries where pharmacists are primarily the first line of contact for patients [21]. This understanding is pivotal to regulations of guidelines, legislations, and action plans towards reduction of antibiotic resistance, a critical issue in public health.

The study findings show that even though most of the pharmacists believe that antibiotic resistance is a worldwide public health issue, and over two-thirds are aware of the Palestinian regulations of proper antibiotic dispensing, around 60% of Palestinian pharmacists may dispense antibiotics without prescription with varying frequency (always, often, and sometimes), which is similar to the global estimate of antibiotic dispensing without prescription [28] and consistent with other Middle Eastern countries [29, 30]. There are numerous recognized factors (patients, business, knowledge, regulations, and so on.) that might contribute to this practice; therefore, there is a need to assess the actual and conceptual performance of pharmacists towards antibiotic resistance.

The key findings of this study demonstrate that pharmacists have an acceptable level of knowledge of antibiotic resistance in terms of general antibiotic uses, mechanisms of antibiotic resistance, and legality of antibiotic dispensing. Most of the study participants agreed that inappropriate use of antibiotics could lead to ineffective treatment, and over two-thirds acknowledged that it's an improper practice for patients to keep leftover antibiotics. However, an alarming key finding is that over 40% of the study participants agreed that upper respiratory tract infections (URTI) should always be treated with antibiotics, which is known in the literature to be mostly caused by viral infection [31]. A recent systematic review demonstrated that URTI is the second most common disease for which pharmacists dispense nonprescription antibiotics [7]. This finding compares favorably with that of Hoxha et al. which reported that only 13% of Albanian pharmacists stated that antibiotics are ineffective against viruses [32]. However, this finding is inconsistent with other studies that indicated pharmacists are knowledgeable of URTI [33], and could lead antimicrobial stewardship programs in URTI management [34]. Therefore, this finding needs further investigation as our study participants have demonstrated higher knowledge of other aspects of antibiotic uses.

On the other hand, the study participants showed a higher level of perceived knowledge of antibiotics and the issue of bacterial resistance, and around one-third of the pharmacists reported that pharmacists' level of knowledge is one of the reasons for selling antibiotics without a prescription. This finding is consistent with a recent study in 30 EU/EEA countries, which has found that most pharmacists agree that they know what antibiotic resistance is [13]. However, this perception of high knowledge could be misleading and lead to improper dispensing practices, as indicated in the Alhomoud et al. study in Saudi Arabia, that pharmacists' self-perception of their knowledge and experience enables them to dispense antibiotics without a prescription [18].

Our study results found a significant difference in the overall level of knowledge according to age and locality, where female and urbanite pharmacists having better knowledge of the matter. A recent scoping review in Southeast Asia has found that in comparison to males, females generally were found to have better knowledge of antibiotics and antibiotic resistance [35]. In addition, Ahmad et al. found that pharmacists residing in the urban areas are more knowledgeable of antibiotic resistance [36]. These findings illustrate the importance of tailoring the antimicrobial stewardship programs to the needs of the pharmacists, considering the sociodemographic differences.

An important observation of this study is the pharmacists' reported reasons for dispensing without a prescription. Over two-thirds of the pharmacists considered the patients' demand and improper use of nonprescription antibiotics of to be a major contributing factor to the issue. Indeed, this finding is consistent with a study in Egypt, which has found that around 55% of the participants believed that patients' personal choice of antibiotic use is one of the main causes of antibiotic resistance [37]. Another study in Hungary deducted that main reason for antibiotic dispensing without prescription is patient demand and a fear of losing customers of the business [38].

Nevertheless, over half of this study pharmacist also reported education of patients on antibiotic uses and indications. Furthermore, they also reported encouraging their patients to get medical consultations and prescriptions. These findings demonstrate the positive attitudes the Palestinian pharmacists have towards antimicrobial resistance. In this study, we have also observed significant differences in both attitudes and practices scores by the educational level and locality. Higher education was more likely associated with better attitudes and practices. A similar finding was observed in a study in Pakistan, in which practices significantly differed between pharmacists with bachelors' and masters' degrees, however, there was no significant difference in perceptions towards antimicrobial stewardship (AMS) [39]. Another study in Thailand found that all of knowledge, attitudes, and practices scores were significantly different between B Pharm and Pharm D degrees [40].

Another key finding of this study is pharmacists' use of the international guidelines for antibiotic dispensing. Less than 20% use the Palestinian General Directorate of Pharmacy's guidelines as a reference for proper dispensing practice. This observation emphasizes the need for diligent regulation and application of regulations that apply in the Palestinian community. Additionally, the majority expressed the willingness to participate in educational programs about antibiotic resistance, mostly as participants, and to a greatly lesser extent, as mentors, developers, and consultants. This finding further emphasizes the pharmacists' perception of their contribution to the problem and their approval of the importance of laws and proper enforcement of legislations. This role is indeed recognized by pharmacists themselves in several studies [20, 41, 42].

Despite these findings, there is a need to emphasize that the issue of antibiotic resistance is not solely the responsibility of pharmacists. Many sectors of the community contribute to the issue, including physicians, veterinarians, dentists, and the public, respectively [43–47]. This implies the role of public awareness of antibiotic resistance, and in the context of this study, this signifies the role of pharmacists in raising public awareness, a multihit approach that might lower the burden of the problem.

The study has been limited by social desirability bias, which we aimed to control through anonymity. Anonymity is considered to lower social anxiety and social desirability bias [48]. Moreover, it was observed that more female pharmacists responded to the survey. This was also similarly observed in other recent surveys [42]. Moreover, many of the responses on the Likert scale questions were uncertain or sometimes, which might decrease the assurance of the actual responses. However, to mitigate this effect, the scales' responses were not summed or recategorized, and the responses were presented as they were originally reported.

## 5. Conclusions

This study aimed to investigate the knowledge, attitudes, and practices of Palestinian pharmacists towards antibiotic resistance. Despite acceptable knowledge of antibiotic resistance and positive attitudes towards the issue, dispensing antibiotic without a prescription is high. Insufficient commitment to local regulations and guidelines were found. The study results showed significant differences in knowledge level by gender and locality and in attitudes and practices by education and locality. An intervention program directed mainly towards practices among pharmacists is imperative in improving antibiotic use and to minimizing the resistance. There is a need for an in-depth analysis of pharmacists' role in antibiotic resistance.

## Figures and Tables

**Figure 1:** Contributing factors to antibiotic resistance.

**Figure 2:** Reasons for dispensing antibiotics without prescription.

**Table 1:** Demographic and professional characteristics of the respondents.

Variable	Category	*N* (%)
*Gender*	Male	73 (48)
	Female	79 (52)

*Age*	<30 years	77 (50.7)
	≥30 years	75 (49.3)

*Years of experience*	<10 years	90 (59.2)
	≥10 years	62 (40.8)

*Locality*	Rural	78 (51.3)
	Urban	74 (48.7)

*Education level*	BPharm	110 (75.3)
	Postgraduate studies	21 (14.4)
	Pharm D	15 (10.3)

*Employment type*	Manager	54 (35.5)
	Employee	98 (64.5)

*Employment status*	Full time	43 (28.3)
	Part time	109 (71.7)

*Total number of employed pharmacists*	1-2	61 (40.1)
	≥3	91 (59.9)

*Number of employed pharmacists working at once*	1	95 (62.5)
	≥2	57 (37.5)

**Table 2:** Knowledge towards antibiotics, antibiotics' uses, legality of antibiotic dispensing, and self-perception of knowledge level.

Question	Disagree		Neutral	Agree	
	SD^*a*^	D^*b*^		A^*c*^	SA^*d*^
	*n* (%)				
*Knowledge about antibiotics and antibiotic use*					
Inappropriate use of antibiotics can lead to ineffective treatment	5 (3.3)	3 (2)	4 (2.6)	28 (18.4)	112 (73.7)
Antibiotics can be used to alleviate pain	44 (28.9)	66 (43.4)	22 (14.5)	12 (7.9)	8 (5.3)
Patients can stop taking antibiotics upon symptoms' improvement	96 (63.2)	35 (23)	8 (5.3)	10 (6.6)	3 (2)
It is considered a good practice to keep leftover antibiotics for similar use in the future	67 (44.1)	34 (22.4)	31 (20.4)	12 (7.9)	8 (5.3)
Upper respiratory infections (URI) should always be treated with antibiotics	10 (6.6)	16 (10.5)	56 (36.8)	57 (37.5)	13 (8.6)
Antibiotics can kill normal flora in the body, thereby causing secondary infections	4 (2.6)	7 (4.6)	51 (33.6)	46 (30.3)	44 (28.9)
Antibiotics can cause allergic reactions	3 (2)	8 (5.3)	15 (9.9)	50 (32.9)	76 (50)
Amoxicillin is an antibiotic	9 (5.9)	5 (3.3)	3 (2)	5 (3.3)	130 (85.5)
Panadol and aspirin are antibiotics	125 (82.2)	8 (5.3)	10 (6.6)	6 (3.9)	3 (2)

*Knowledge about antibiotic resistance*					
Prescribing broad-spectrum antibiotics is always better even if there are narrower spectrum antibiotics that are effective	52 (34.2)	25 (16.4)	11 (7.2)	24 (15.8)	40 (26.3)
The mechanism of resistance to beta-lactams in *Klbesiella pneumoniae* is mainly enzymatic	6 (3.9)	8 (5.3)	30 (19.7)	53 (34.9)	55 (36.2)
The mechanism of resistance to vancomycin-resistant *Enterococcus faecalis* is alteration of binding sites	9 (5.9)	14 (9.2)	64 (42.1)	50 (32.9)	15 (9.9)
Wrong choice of antibiotics may lead a pathogen to lose its sensitivity towards a specific antibiotic	4 (2.6)	31 (20.4)	19 (12.5)	28 (18.4)	70 (46.1)
Forgetting one or two doses of an antibiotic does not contribute to antibiotic resistance	47 (30.9)	58 (38.2)	20 (13.2)	20 (13.2)	7 (4.6)
Resistant bacterial strains could not be spread in healthcare facilities	34 (22.4)	26 (17.1)	39 (25.7)	40 (26.3)	13 (8.6)
*Knowledge about the legality of antibiotic dispensing*					
I am not familiar with the legislations concerning dispensing antibiotics (with or without a prescription) in the west bank	68 (44.7)	31 (20.4)	25 (16.4)	17 (11.2)	11 (7.2)
In the west bank, antibiotics are categorized under prescription drugs	10 (6.6)	19 (12.5)	11 (7.2)	37 (24.3)	75 (49.3)

*Self-perception of knowledge level*					
My knowledge regarding the pharmacological aspects of antibiotic therapy is appropriate	4 (2.6)	11 (7.2)	28 (18.4)	55 (36.2)	54 (35.5)
My knowledge regarding bacterial resistance is appropriate	2 (1.3)	22 (14.5)	47 (30.9)	54 (35.5)	27 (17.8)

^*a*^SD: strongly disagree. ^*b*^D: disagree ^*c*^SA: strongly agree. ^*d*^A: agree.

**Table 3:** Attitudes towards antibiotic resistance (AR) and guidelines of antibiotic dispensing.

Question	Disagree		Neutral	Agree	
	SD^*a*^	D^*b*^		A^*c*^	SA^*d*^
	*n* (%)				
Antibiotic resistance is an important and serious public health issue facing the world	2 (1.3)	11 (7.2)	24 (15.8)	49 (32.2)	66 (43.4)
Dispensing antibiotics without prescription is a common practice among community pharmacists in the West Bank	6 (3.9)	12 (7.9)	55 (36.2)	43 (28.3)	36 (23.7)
Patient personal choice of antibiotic use and overuse could contribute to antibiotic resistance	6 (3.9)	5 (3.3)	24 (15.8)	35 (23)	82 (53.9)
It obligatory for me to educate and inform patients requesting antibiotics without a prescription and are probably not in need of antibiotic therapy	7 (4.6)	24 (15.8)	24 (15.8)	37 (24.3)	60 (39.5)
Relevant conferences, workshops, and other educational activity are required to be attended by community pharmacists to enhance understanding of antimicrobial stewardship	1 (0.7)	12 (7.9)	32 (21.1)	49 (32.2)	58 (38.2)
The development of local guidelines would be more useful than the international ones for antimicrobial resistance	4 (2.6)	12 (7.9)	56 (36.8)	56 (36.8)	24 (15.8)

^*a*^SD: strongly disagree. ^*b*^D: disagree. ^*c*^SA: strongly agree. ^*d*^A: agree.

**Table 4:** The number and percentage of antibiotics dispensed and demanded per pharmacy per day.

The number of antibiotics:	≤20	>20	Didn't answer
	*n* (%)		
Dispensed antibiotics per day	87 (57.2)	59 (38.8)	6 (3.9)
Dispensed antibiotics with prescription per day	118 (77.6)	29 (19.1)	5 (3.3)
Demanded antibiotics without prescription per day	138 (90.8)	8 (5.3)	6 (3.9)

**Table 5:** Practices of pharmacists towards antibiotic dispensing and resistance.

Question	Always	Often	Sometimes	Rarely	Never
	*n* (%)				
I dispense antibiotics without prescription upon patient request	40 (26.3)	13 (8.6)	38 (25)	33 (21.7)	28 (18.4)
I dispense antibiotics without prescription for adult patients with minor bacterial infections	4 (2.6)	45 (29.6)	56 (36.8)	25 (16.4)	22 (14.5)
I encourage patients to obtain a physician's consult and prescription	57 (37.5)	34 (22.4)	39 (25.7)	20 (13.2)	2 (1.3)
When dispensing antibiotics, I enquire about any known drug allergies or health problems	85 (55.9)	18 (11.8)	32 (21.1)	14 (9.2)	3 (2)
When dispensing antibiotics without prescription, I warn about their potential adverse effects	45 (29.6)	27 (17.8)	36 (23.7)	34 (22.4)	10 (6.6)
When dispensing antibiotics without prescription, I inform patients about the significance of adhering and completing the full course of an antibiotic	54 (35.5)	34 (22.4)	23 (15.1)	32 (21.1)	9 (5.9)
I dispense antibiotics without prescription on the patient's request for a familiar patient	33 (21.7)	23 (15.1)	45 (29.6)	27 (17.8)	24 (15.8)
I seek additional clinical information (e.g., drug interaction, ADRs, allergy) before deciding to dispense antibiotics without a prescription	25 (16.4)	31 (20.4)	45 (29.6)	29 (19.1)	22 (14.5)

**Table 6:** Regression analyses of potential sociodemographic determinants association with knowledge, attitudes, and practices' scores.

Variable	Knowledge				Attitudes				Practices			
	OR	SE	95% CI	*p* value	OR	SE	95% CI	*p* value	OR	SE	95% CI	*p* value
Gender	1.23	1.82	(0.94, 8.15)	0.014	1.10	0.78	(0, 2.32)	0.322	1.12	1.38	(0, 4.53)	0.191
# of employed pharmacists	0.76	1.78	(−9.7, −2.67)	0.001	1.02	0.76	(0, 1.67)	0.823	0.74	1.34	(−7.72, −2.42)	0.001
# of employed pharmacists working at once	0.97	1.79	(0, 2.93)	0.736	1.03	0.76	(0, 1.72)	0.779	1.06	1.35	(0, 3.58)	0.498
Education	0.98	1.24	(0, 2.15)	0.807	1.15	0.53	(0, 1.87)	0.123	1.10	0.94	(0, 3.06)	0.198
Employment type	1.05	1.94	(0, 5.03)	0.540	1.02	0.83	(0, 1.77)	0.872	1.01	1.46	(0, 3.05)	0.919
Age	1.03	2.68	(0, 6)	0.792	1.17	1.14	(0, 3.52)	0.274	0.82	2.02	(0, 0.84)	0.121
Years of experience	1.00	2.94	(0, 5.86)	0.988	0.96	1.26	(0, 2.13)	0.776	1.14	2.22	(0, 6.53)	0.337
Locality	1.55	1.59	(6.39, 12.66)	0.001	1.08	0.68	(0, 1.98)	0.344	1.50	1.20	(4.29, 9.02)	0.001

## Data Availability

The authors confirm that the data supporting the findings of this study are available within this article. Raw data that support the findings of this study are available from the corresponding author, upon reasonable request.
